# Automatic Gray Image Coloring Method Based on Convolutional Network

**DOI:** 10.1155/2022/5273698

**Published:** 2022-04-26

**Authors:** Jiayi Fan, Wentao Xie, Tiantian Ge

**Affiliations:** Suzhou Institute of Technology, Jiangsu University of Science and Technology, Zhangjiagang, Jiangsu 215600, China

## Abstract

Image coloring is a time-consuming and laborious work. For a work, color collocation is an important factor to determine its quality. Therefore, automatic image coloring is a topic with great research significance and application value. With the development of computer hardware, deep learning technology has achieved satisfactory results in the field of automatic coloring. According to the source of color information, this paper can divide automatic coloring methods into three types: image coloring based on prior knowledge, image coloring based on reference pictures, and interactive coloring. The coloring method can meet the needs of most users, but there are disadvantages such as users cannot get the multiple objects in a picture of different reference graph coloring. Aiming at this problem, based on the instance of color image segmentation and image fusion technology, the use of deep learning is proposed to implement regional mixed color more and master the method. It can be divided into foreground color based on reference picture and background color based on prior knowledge. In order to identify multiple objects and background areas in the image and fuse the final coloring results together, a method of image coloring based on CNN is proposed in this paper. Firstly, CNN is used to extract their semantic information, respectively. According to the extractive semantic information, the color of the designated area of the reference image is transferred to the designated area of the grayscale image. During the transformation, images combined with semantic information are input into CNN model to obtain the content feature map of grayscale image and the style feature map of reference image. Then, a random noise map is iterated to make the noise map approach the content feature map as a whole and the specific target region approach the designated area of the style feature map. Experimental results show that the proposed method has good effect on image coloring and has great advantages in network volume and coloring effect.

## 1. Introduction

With the emergence of digital media technology and the popularity of the Internet, the animation industry has been greatly developed and advanced [1–3]. Animation works usually have two forms of expression, two-dimensional animation and three-dimensional animation, among which two-dimensional animation works have strong representation, character drawing and coloring are more natural, and three-dimensional animation works are not limited by the physical engine. At present, two-dimensional animation works still have a wide influence. Generally, ordinary animation video requires at least 25 frames per second to ensure the continuity of the video, while a 25-minute animation video requires 37,500 frames of images [4, 5]. Although the drawing of intermediate frames can be made according to the reference of key frames, the heavy task still requires the cooperation of multiple workers. In addition, after the middle frame line draft image is completed by the ordinary painter, it should be checked and modified by the animation instructor to maintain the consistency of the middle frame action and color and ensure the continuous effect of the character action in the line draft video [6]. Therefore, the research on the coloring and auxiliary rendering of animation line draft image can not only help the new artist to improve the drawing efficiency but also to reduce the manpower and material resources required for drawing line draft and coloring. In general, the key frame usually refers to the first and last frame of the animation shot. The post-production mainly completes the synthesis of characters and backgrounds, the addition of light and shadow effects, and the work of film editing and dubbing [7, 8].

Coloring is a very important stage after animation line draft image creation, time-consuming, and tedious; current cartoon makers will adopt some business equipment and software speed line art image color work but did not greatly improve production efficiency.In these papers, a new automatic coloring method for line art images is proposed based on the reference of color images, and the method is extended to similar color areas [9–12]. Inspired by the successful application of generative models in image synthesis tasks in recent years, the researchers use deep convolutional neural networks (DCNNs) and put forward many methods for automatic coloring of line draft images, but the coloring results of these methods are not controllable and often accompanied by color artifacts. In recent years, thanks to the prosperity of Internet technology, digital media industry has also become the core industry of the 21st century knowledge economy, such as film and television advertising online games, and a film and television work or an online game to attract people's attention often needs a dazzling poster [13–15]. Good works are not only reflected in content design but also in color collocation. Whether for the creation of pictures or videos, colorization is an extremely important link. However, this is not an easy task; the choice and collocation of color are a test of the artist's artistic foundation and time-consuming. Moreover, for a good work that has been created, if the color of one of the objects is not satisfied with the need to recolor, the existing method is direct gray recolor, which is a huge project. Therefore, the multiarea coloring of images is a significant research work for both academia and industry [16, 17].

Convolutional neural network is a simple and efficient network completely different from previous deep learning models. General deep learning models contain an overall neural network, but CNN breaks this structural mode. It consists of two subnetworks, namely, generator subnetwork and discriminator subnetwork. The generator can be used to extract image features and generate false images. Discriminators can be used to discriminate between real and fake images, giving a probability to conclude that the image is more likely to be real or to generate a fake image. In this process, both the generator model and the discriminator model are constantly trained [18]. With the increase in iteration times, the generator model's false image forgery ability becomes stronger and stronger, and the discriminator's accurate identification ability of true and false images becomes stronger and stronger and finally tends to converge. Therefore, the CNN model is widely used in image processing and is one of the most commonly used models in the field of image coloring [19–22].

## 2. Related Works

An et al. [23] asked users to draw a color curve for graffiti and set the gradient range of the curve to control the spread of graffiti. Specifically, the method takes a set of diffusion curves as constraints and obtains the final image by solving Poisson's equation. However, all the above methods require a lot of manual interaction to achieve target coloring. In order to reduce the manual work and realize the specified color style coloring, researchers proposed a coloring method based on reference image. JWA et al. [24] used graph structure to represent the relationship between different regions of line draft image and solved the matching problem through quadratic programming. However, complex line draft image is usually difficult to be accurately segmented, and the same semantic region will be divided into multiple blocks. At present, researchers have proposed line draft map guided by reference image based on the deep learning image coloring method which avoids the requirement of image segmentation accuracy. Chen et al. [25] used conditional generative adversarial networks (cGANs) to color grayscale images without requiring users to interactively fine-tune the coloring results. However, this method is only suitable for learning the relationship between grayscale and color image, not line image. Active learning framework learns domain classification labels in small data sets and helps users to select the data to be labeled in unlabeled sets, so as to continuously update the learning model parameters and improve the accuracy of the model for unlabeled region classification labels. Zeng et al. [26] proposed an adaptive active learning method, which combined information density calculation with least uncertainty calculation to select marked instances, different from previous methods of selecting marked data based on uncertainty. Farid et al. [27] proposed the coloring task which involves specifying a three-dimensional information, such as RGB channel, from the one-dimensional information of grayscale image, that is, intensity or brightness. The mapping between the one-dimensional information and three-dimensional information is not unique. Colorization is ambiguous in nature, and appropriate external information needs to be provided. Therefore, the coloring algorithm based on image brightness weighted color mixing and fast feature space distance calculation can achieve high quality static image at the cost of a small part of the calculation cost and improve the speed of the algorithm.

Kotecha et al. [28] trained an automatic system for colorization of black and white images and trained the model to predict the color information of every pixel in the black and white images by using deep network to learn the detailed features of the color images. Berger et al. [29] proposed a new automatic coloring method for comics. Image features include global features and local features. Global features include the overall outline of the image, while local features include some details of the image. Based on convolutional neural network, the network contains two subnetworks, local feature extraction network and global feature extraction network, in order to achieve the purpose of cartoon image processing at any resolution. In recent years, with the popularity of deep learning, the mainstream of cartoon coloring gradually developed is to use two different methods to realize simple coloring algorithm and deep learning model. Among the methods based on deep learning, a variety of deep learning models have been used to complete the task of image translation. Many researchers have tried to use human intelligence to solve the task of automatic coloring of pictures. A Thakur et al. [30] pointed out that there are few papers on image processing using unsupervised learning CNNs network, so they proposed DCGAN, a deep volume network, to realize CNN's attempts in supervised learning and unsupervised learning, respectively. How to accurately cut the image region is also a major factor affecting the final image color accuracy and quality; for image region segmentation, many researchers have done related research. Oladi et al. [31] decided to consider not only adjacent pixels with similar intensity but also distant pixels with the same texture, so they combined the two to enhance the visual effect. Through experiments, they found that better results can be obtained when coloring pixels near edges based on texture similarity and pixels in smooth regions based on intensity similarity. The method can also be used to color comics, and they have developed a set of interface tools that allow users to tag and color and modify target images. Qiao et al. [32] implemented two coloring methods based on U-NET. The main innovations of this method are as follows: one is to train a deep neural network to directly predict the mapping from grayscale images with colored points to color images; second, the network will also provide users with a data-driven color palette, suggesting the ideal color of the gray map in a given location. This approach can also bring the benefit of reducing the workload for users, and it can also calculate the global histogram of a color reference map to color the gray map [10, 33].

From the above analysis, we know that the above methods have studied the automatic gray image coloring widely. However, some problem still exists. For example, no scholar has applied the CNN model to this field till now, so the research here is still a blank, which has great theoretical research and practical application value for logistics enterprises [34].

This paper consists of five parts. The first and second parts give the research status and background. The third part is the automatic gray image coloring by the CNN model. The fourth part shows the experimental results. The experimental results of this paper are introduced and compared and analyzed with relevant comparison algorithms. Finally, the fifth part gives the conclusion of this paper.

## 3. Automatic Gray Image Coloring by CNN Model

### 3.1. The Process of Automatic Gray Image Coloring

For any enterprise, capital is the source of its life; financing is a way to revitalize the enterprise capital, improve the effective utilization rate of capital, and obtain profits. With the modern new production organization mode—the new financing mode produced by supply chain—supply chain finance financing has become a hot spot, supply chain finance is called the general trend, and enterprises must have its reasons and conditions for supply chain finance financing. As a result, those with the greatest impact of stress and the greatest capacity to take the most drastic and effective action for change are the most likely to achieve the best performance. This paper will establish the supply chain financial performance evaluation index system of warehousing and logistics enterprises from the four dimensions of pressure dimension, action dimension, ability dimension, and driving factor dimension. The whole system of the method is given in Figure 1.

Except for the CNN model, VGG network achieved good results in ILSVRC positioning and classification tasks, respectively. VGG network inherited the main convolution-pooling network in AlexNet. They abandoned large convolution kernels and replaced them with multiple convolution kernels with a size of 3 × 3, which could reduce the number of network parameters and increase the network depth. This can be said to be the in-depth version of AlexNet; deeper network better fits complex nonlinear problems. Even so, the number of VGG network parameters is still very large.Generally speaking, a VGG network contains 500 parameters, so the model takes up a lot of storage space. However, thanks to its excellent feature extraction ability, it is very suitable for the auxiliary task of feature extraction in some image processing tasks. Differential network does not refer to a specific network, but a structure that can be used in any network model. Residual structure is a connection mode that prevents network degradation through a hop connection. In addition, even with the use of ReLU activation function, the phenomenon of gradient disappearance will occur with the increase in the number of network layers, while the residual structure can solve the above problems. The residual structure adopts the method of skip connection in the network structure. In conclusion, the CNN model shows better performance than the VGG network; hence, the CNN is selected in this paper.

### 3.2. Convolutional Neural Network

In the process of image processing, we often use matrix convolution to calculate the feature of image. There are two types of matrix convolution: full convolution and valid convolution. The definition of full convolution is as follows:

(1) $$\begin{array}{c} z\left(u,v\right)=\sum_{i=-\infty }^{\infty }\sum_{j=-\infty }^{\infty }x_{i,j}\cdot k_{u-i,v-j},\\ \sigma_{t}^{2}=\alpha_{0}+\sum_{i=1}^{p}\alpha_{i}a_{t-i}^{2}+\sum_{q}^{j=1}\beta_{j}\sigma_{t-j}^{2}. \end{array}$$

Assuming that *X* is the m-order matrix and *k* is the *n*-order matrix, the definition of effective convolution is

(2) $$\begin{array}{c} z\left(u,v\right)=\sum_{i=-\infty }^{\infty }\sum_{j=-\infty }^{\infty }x_{i+u,j+v}\cdot k_{roti,j}\cdot \chi \left(i,j\right). \end{array}$$

Assume that

(3) $$\begin{array}{c} \chi \left(i,j\right)=0\text{ or }1\text{.} \end{array}$$

Convolution layer (the previous layer is the input layer): in the convolution, the data is input to the input layer in 3d form, and then the convolution kernel of the first layer and the corresponding functional module convolve the input data. We add a bias term to each output, and the output of the convolution layer is as follows:

(4) $$\begin{array}{c} z_{u,v}^{\left(l\right)}=\sum_{i=-\infty }^{\infty }\sum_{j=-\infty }^{\infty }x_{i+u,j+v}^{\left(l-1\right)}\cdot k_{rot}^{\left(l\right),j}\cdot \chi \left(i,j\right)+b^{\left(l\right)},\\ \chi \left(i,j\right)=0\text{ or }1,\\ a_{u,v}^{\left(l\right)}=f\left(z_{u,v}^{\left(l\right)}\right). \end{array}$$

To ensure that variance is positive, that is, variance exists and is finite as follows:

(5) $$\begin{array}{c} \sum_{i=1}^{\max\left(p,q\right)}\left(\alpha_{i}+\beta_{i}\right)<1. \end{array}$$

After the input feature graph passes through the convolution layer, we get its feature graph. Now, we hope to use these feature graphs to train the classifier. Theoretically, we can use all the extracted feature graphs to train the classifier. In order to solve this problem, we can use the aggregation of the statistical method. For example, we can replace all the original features with the average of the image features, which is faster and less prone to over-fitting than all the features used. So, this aggregation is called pooling, and pooling is divided into average pooling and max pooling. Here, we take the average pooling method as an example and use the weight of each unit of the convolution kernel. After each convolution operation, a bias unit is still added. The output of the subsampling layer is as follows:

(6) $$\begin{array}{c} z_{i,j}^{\left(l+1\right)}=\beta^{\left(l+1\right)}\sum_{u=ir}^{\left(i+1\right)r-1}\sum_{v=jr}^{\left(j+1\right)r-1}a_{u,v}^{\left(l\right)}+b^{\left(l+1\right)},\\ a_{i,j}^{\left(l+1\right)}=f\left(z_{i,j}^{\left(l+1\right)}\right),\\ K_{a}^{\phi }=\frac{3-3{\left(\alpha_{1}+\beta_{1}\right)}^{2}}{1-2\alpha_{1}^{2}-{\left(\alpha_{1}+\beta_{1}\right)}^{2}}-3. \end{array}$$

If the subsampling layer is followed by the convolution layer, the calculation method is the same as that described by the multilayer neural network, and the output is as follows:

(7) $$\begin{array}{c} z_{u,v}^{\left(l+2\right)}=\sum_{i=-\infty }^{\infty }\sum_{j=-\infty }^{\infty }a_{i+u,j+v}^{\left(l+1\right)}\cdot k_{i,j}^{\left(l+2\right)}\cdot \chi \left(i,j\right)+b^{\left(l+2\right)},\\ a_{u,v}^{\left(l+2\right)}=f\left(z_{u,v}^{\left(l+2\right)}\right). \end{array}$$

The schematic diagram of a typical convolutional neural network is shown in Figure 2:

## 4. Experimental Results and Analysis

### 4.1. Introduction to Experimental Environment and Data Set

This line of business on Windows 10 OS runs a HMP RTX 2070S 8 GB video memory, AMD Ryzen 2400G CPU, 16 GB DDR4 software environment: Deep learning framework Pytorch 1.8. Python 3.7 CUDA 10.0 data set uses Place 365 outdoor landscape, including buildings, cabins, landscapes, courtyards, and more than 50 categories. The Epoch is 10. The comparison algorithm is trained by a business line with the same data set, and the Epoch trained is also 10.

In this experiment, the initial learning rate is set to 0.02 by experience, the attenuation weight coefficient is 0.0001, the updated weight is 0.1, the updated weight attenuation system is 0.0002, the maximum number of iterations is 10000, epoch is 600 times, and the random gradient descent method Batch is selected. Batch training options are 50.

### 4.2. Experimental Results Analysis

Firstly, the comparison of the results of the real standard foreground coloring using random noise graph and image conversion network, respectively, includes the comparison of its coloring efficiency, and then the two foreground coloring methods, respectively, combined with U-NET and Poisson fusion, are shown to achieve the whole picture coloring. And the multiregion color rendering method based on random generated noise graph and basis forward transformation network is proposed, respectively.  Figure 3 shows the coloring effects of different categories of images.

Transformation of regional colours is possible in random noise images and image transformation networks, but there are massive differences between the two speeds and the colours of the ginseng, and each colour needs to be trained, while the image transformation network taken is made up of cyclic transformations. The network generates the noise graph, then updates the parameters of the image conversion network training, and saves the optimal solution.

When one or more shells appear in the picture, you can select a different reference image for each earmark in the picture and color all ICONS in the picture at the same time by selecting the reference image. According to the input semantic map of gray image, one or more marks in the image are colored. In addition, due to the addition of semantic information as a strong constraint condition, the two color labeling methods in this paper have stronger constraints, so as to obtain better graphic coloring effect.  Figure 4 shows the coloring results of the same and different categories, which can make the coloring results more diverse and conducive to the user's image creation. The results show the combination of foreground coloring, back coloring, and Poisson melting.

It can be seen that the simple fusion effect directly depends on the result of image instance segmentation, and the quality of the result of instance segmentation determines the fusion effect. However, the current instance segmentation technology can only circle the general target, and there is still a lack of edge processing. Therefore, this paper uses the CNN algorithm to fuse the background and foreground after coloring, so that the edge can smoothly transition.

Because the final effect of coloring is difficult to measure with mathematical way, the richer the color, the greater the final loss, but the final effect is acceptable. Figures 5 and 6 show the comparison of some experimental effects.  Figure 6 shows the recoloring effect of color photos, and Figure 6 shows the coloring effect of black and white photos. From the perspective of recoloring effect of color images, the images colored by the proposed method are more colorful and have better processing of details and light and shadow effects than other algorithms. DCGAN's effect is always dark, and the algorithm in this paper does not recognize the ground in group *E*, but other groups of images have relatively good effects.

In the colorful image coloring shown in Figure 5, the method presented in this paper has good semantic properties, vivid colors, and good restoration of sky. The BP algorithm is also good in general, but the restoration of sky is not accurate, and RNN is dull. The algorithm in this paper has a better coloring effect at the gap between leaves and sky and is more accurate in coloring buildings, while the BP algorithm is green. The proposed algorithm is relatively accurate to color the ground, while the BP algorithm may treat the map as the ocean. The coloring effect of several groups of results of the RNN algorithm is too dull.

As shown in Figure 6, it can be seen from the comparison with the original picture that the color of CNN model proposed in this paper is more realistic and natural; that is to say, this paper has obtained the best image coloring effect. .

As shown in Figure 7, just add some color prompt graffiti lines to each part of the scene, and the model can render other uncolored parts in the image area according to the prompts. Moreover, this color rendering is not pure color filling. The transition of light and dark colors makes the whole coloring effect more natural and not rigid. For example, in the pictures of the second group of buildings, only a pure blue graffiti hint line is given instead of a pure color. However, the interaction between colors is not very obvious there are some rise in space, such as in the first set of interaction diagrams had two yellow graffiti decorate tip lines, in addition to other part is not in the yellow line, but the generated version of athletes central sleeve are also be rendered into yellow, with the expected painting effect exists some gap. However, MSE generally showed a downward trend.

Figure 8 shows the effect comparison before and after color refinement. In the CNN algorithm, each gray pixel performs full-image search and matching, and the pixel with the smallest error is selected in the source image for matching. Therefore, all pixels in the target image should be able to find matching pixels in the source image. However, we are still unable to obtain a very satisfactory method for both color quality and color speed. How to make before and after color refinement achieve a win-win situation is the ultimate goal of this study. In terms of improving quality, more and more matching guiding factors have been proposed, instead of relying only on the brightness mean and brightness variance as the only criteria for matching search. For example, the slope and kurtosis containing nonlinear properties of images can guide pixel matching. In order to improve the speed, the tree structure is used to classify pixels as much as possible, so that the matching process has a clear goal, rather than blindly carrying out full image search.

## 5. Conclusions

In recent years, with the vigorous development of computer hardware equipment, artificial intelligence has appeared more and more frequently in people's vision. The image automatic color not only can increase the interest in everyday life but also can improve the efficiency of some work, such as poster making, etc. So, the gray image coloring technology has also attracted the attention of many researchers. In this article through the large number of literatures, the survey found existing in coloring technology can meet the needs of most of the color but still exist with some disadvantages, such as not to picture one or more specific areas in color and not only change the image of one or more specific areas in color. Aiming at these deficiencies, this paper uses semantic and image fusion technology to realize the image segmentation of regional color more, separately from the multiple target and the background color of the image. Background coloring is carried out end-to-end coloring by CNN, while target coloring needs to be colored according to the color reference graph. Target coloring is divided into two coloring methods, one is iterative image coloring and the other is training image conversion.

Gray image automatically chromatically is an important research direction in the field of image . With the continuous development of deep learning in recent years, automatic coloring of gray image is gradually realized based on the deep learning model. The simple coloring algorithm is generally inferior to the deep learning model. Both interactive coloring reference coloring and automatic coloring can be realized by deep learning. However, there are still some limitations in using deep learning to complete the gray image automatic coloring task; for example, the color effect learning is not in place, the gray image line contour recognition is not accurate evaluation method and is not unified, and there is no inclusive professional gray image coloring platform and so on.

Using the color based on classification of network, this paper proposes a new CNN network using a traditional Gaussian convolution encoder and a hollow convolution stack structure to perform automatic coloring of gray images. Compared with the results of other business methods, it has advantages in the final coloring effect and volume control.

## Figures and Tables

**Figure 1:** The framework and flow chart of the proposed method.

**Figure 2:** The schematic diagram of convolutional neural network.

**Figure 3:** Coloring results for different categories of images.

**Figure 4:** Category at the same time color result comparison.

**Figure 5:** Different methods for recoloring color pictures.

**Figure 6:** Different methods for recoloring gray image.

**Figure 7:** The error curves of different scenes by CNN.

**Figure 8:** Effect comparison before and after color refinement.

## Data Availability

The dataset can be accessed upon request.
